The article "High-Resolution Histopathological Image Classification Model Based on Fused Heterogeneous Networks with Self-Supervised Feature Representation" was published in 2022. Journal: Biomed Res Int.

# High-Resolution Histopathological Image Classification Model Based on Fused Heterogeneous Networks with Self-Supervised Feature Representation

**DOI:** 10.1155/2022/8007713

**Published:** 2022-08-21

**Authors:** Zhi-Fei Lai, Gang Zhang, Xiao-Bo Zhang, Hong-Tao Liu

**Affiliations:** ^1^Information Engineering College, Guangzhou Panyu Polytechnic, Guangzhou 511483, China; ^2^School of Automation, Guangdong University of Technology, Guangzhou 510006, China

## Abstract

Applying machine learning technology to automatic image analysis and auxiliary diagnosis of whole slide image (WSI) may help to improve the efficiency, objectivity, and consistency of pathological diagnosis. Due to its extremely high resolution, it is still a great challenge to directly process WSI through deep neural networks. In this paper, we propose a novel model for the task of classification of WSIs. The model is composed of two parts. The first part is a self-supervised encoding network with a UNet-like architecture. Each patch from a WSI is encoded as a compressed latent representation. These features are placed according to their corresponding patch's original location in WSI, forming a feature cube. The second part is a classification network fused by 4 famous network blocks with heterogeneous architectures, with feature cube as input. Our model effectively expresses the feature and preserves location information of each patch. The fused network integrates heterogeneous features generated by different networks which yields robust classification results. The model is evaluated on two public datasets with comparison to baseline models. The evaluation results show the effectiveness of the proposed model.

## 1. Introduction

Histopathological images are the imaging of tissue sections under a microscope, and numerous studies have validated and demonstrated their value in biomedical research [1–3]. Compared with other medical imaging modalities, histopathological images contain a higher degree of information density, and an image can contain elements such as nuclei, cells, tissues, and stroma that are different in structure and texture. With the advancement of imaging and image processing equipment, whole slide image (WSI) is widely used in computer-aided systems for pathological diagnosis [4, 5]. WSI retains a large amount of detailed information of tissue sections, provides strong support for the identification of pathological characteristics and diagnosis of lesions [6], and is in fact the gold standard for the diagnosis of many cancers.

However, it is still a great challenge to directly process WSI through deep neural networks due to its extremely high resolution. For example, in the TCGA database [7], a WSI (entity ID: TCGA-HT-768101Z-00-DX4) in SVS format in the TCGA-HT subset has a size of 666 MB with resolution 79679∗64810. Limited by the computing power of computer hardware, it is difficult to directly apply deep neural network for analysis of such high-resolution images [8]. There are currently two main approaches to solve this problem. The first one is to reduce the resolution of WSI so that it can be efficiently processed by deep learning models. However, reducing the resolution will lead to a great loss of information in WSI, which will lead to a decrease in the accuracy of the model, especially in tasks such as cell nucleus identification and tissue structure classification that need to be analyzed by pixel-level features [9–11].

The article "High-Resolution Histopathological Image Classification Model Based on Fused Heterogeneous Networks with Self-Supervised Feature Representation" was published in 2022. Journal: Biomed Res Int.

The second method follows the idea of divide and conquer. First, the WSI is divided into patches, and the resolution of each patch is small enough to be input to the deep learning model for training and feature extraction, and then, the features of these patches are fused and fed to the analysis model associated with the target task for processing. Huang and Chung [12] proposed an automatic classification model for WSI. They developed a deep model to fuse the features of each patch and preserve their spatial relative positional relationship. The fusion network consists of several fully connected layers with dropout. Wang et al. [13] proposed a system based on deep learning that can detect malignant melanoma in WSIs of eyelid. The method first trained a convolutional neural network to predict the malignant probability of a patch, and then, a heatmap is generated by embedding the malignant probability of each patch into the original WSI. Finally, a random forest is applied to the generated heatmap to obtain the WSI level classification. However, the method requires patch-level labeling, which usually requires a lot of human efforts, and thus has limited applicability. Brancati et al. [14] proposed a deep learning model for WSI classification and scoring. A pretrained ResNet is used as a patch-level feature extractor. The extracted patch features are stacked together based on their spatial information to form a grid-based feature map. Then, an attention model with min and max pooling operations is applied to the feature map to obtain feature vector for final classification. We argue that the attention model with min and max pooling operations is limited in their feature diversity when generating the final classification feature vector. Lai et al. [15] proposed a method for automated grey matter and white matter in WSIs. The method utilized a self-supervised patch encoder and a semisupervised classification model for patch classification. The patch encoder trained on a self-supervised manner is an effective means in label-free model pretraining.

The article "High-Resolution Histopathological Image Classification Model Based on Fused Heterogeneous Networks with Self-Supervised Feature Representation" was published in 2022. Journal: Biomed Res Int.

Recently, the research on WSI analysis model based on deep learning mainly focuses on two key issues. The first is to obtain a compact representation of patches with minimal information loss [16–18]. The second is the fusion of patch features, through which feature vectors or feature maps are obtained for target model training [19, 20]. Our proposed model follows the idea of patch-based WSI analysis method and solves the above two key problems by introducing self-supervised learning [21] and heterogeneous feature fusion mechanism. We use a UNet-based model [22–24] for patch feature representation. The network consists of an encoder (*f*) and a decoder (*h*), and a compact feature vector (*v*) connects them. The training process does not need to consider the label of the image but only needs to make the input and output of the network as close as possible, which can be evaluated by a pixel-wise loss function. Given a set of images *D* = {*I*_0_, *I*_1_, ⋯, *I*_*n*_}, the feature representation model solves the following problem as shown in

(1) $$\begin{array}{c} \arg\underset{f,h}{\min}L\left(h\left(f\left(d\right)\right),D\right), \end{array}$$

where *L* is a pixel-wise loss function evaluating the total difference between the recovery images *h*(*f*(*d*)) and the groundtruth images *D*. The compact feature representation of an input image *I*_*x*_ is *v* = *f*(*I*_*x*_) obtained by minizing the training loss. Note that *f* acts as an encoder to find the optimal feature representation of the input sample and does not contradict the degree of compression of the feature representation. The success of models such as UNet has fully demonstrated that both can achieve better results in an optimization process.

In order to make full use of the different information implied in the image feature expression, we propose to apply deep models with different structures to process *v* parallelly and finally fuse the results together. Four famous deep learning model architectures are considered in this work, i.e., GoogleNet [25–27], VGGNet [28], ResNet [29], and DenseNet [30]. The motivation of applying these four networks with different architectures lies in the aim of obtaining the feature maps with diversity, so as to obtain a more robust analysis model by using the strategy of ensemble learning. The concepts of these deep neural networks are different, and the connection patterns between the processing blocks are also quite different, which makes the extracted depth features diverse. The inception block in GoogleNet makes use of the Network in Network (NiN) [31] structure to obtain different receptive fields. ResNet retains a certain percentage of the output of the previous network layer through the residual module to avoid gradient disappearance. The basic idea of DenseNet is almost the same as that of ResNet. It establishes connections between each pair of layers to make full use of depth features.

The article "High-Resolution Histopathological Image Classification Model Based on Fused Heterogeneous Networks with Self-Supervised Feature Representation" was published in 2022. Journal: Biomed Res Int.

The four subnetworks are placed into a global network with consistent training strategy and loss function, in which the extracted features are fused together. By fusing the feature maps with diversity, features with stronger expressive power can be formed. We briefly explain the motivation for doing so. The traditional ensemble learning method is generally to vote for the output results of classifiers by majority [32]. This is because the performance of traditional classifiers is not so strong, and only differentiated classifier parameters or training sets can be used, so that classifiers can complement each other. However, the deep neural network has strong enough classification ability, and the effect of differentiation is limited. Heterogeneous feature expression is more helpful to improve the effect of the target model.

The main contributions of this work are twofold:

- We propose a self-supervised encoding network for patch feature representation in a WSI. The encoding network can effectively process patches of a WSI while keeping their spatial information, and it can work in a transfer learning pattern
- We propose a classification model which fuses blocks of 4 heterogeneous structures and achieve significant improvement of performance compared to single structures

The remainder of this paper is organized as follows: Section 2 presents the details of the proposed model including the UNet-based self-supervised feature representation method and heterogeneous network-based feature fusion model. The evaluation methods and results are reported in Section 3 followed by a discussion. Finally, we conclude the paper in Section 4.

## 2. Method

### 2.1. Framework

The model proposed in this paper is divided into two parts. The first part is a self-supervised feature extractor (SSFE) based on UNet, which extracts compact features of the input WSI patches and compresses the features while keeping the patch information as much as possible. The second part is a heterogeneous feature fusion model (HFFM), which uses four different network blocks to convolve, pool, and activate the patch feature cube nonlinearly to get the feature vectors for target analysis tasks. The two parts are connected by the feature cube obtained by patch feature stacking.  Figure 1 sketches the main framework of the proposed model.

The article "High-Resolution Histopathological Image Classification Model Based on Fused Heterogeneous Networks with Self-Supervised Feature Representation" was published in 2022. Journal: Biomed Res Int.

The two parts of the model are trained separately. For SSFE, its main goal is to get a compact feature representation of the patch through training, which is realized by a network with basically symmetrical structure. The input patch is downsampled and upsampled for the same number of times, and the difference between the input patch and the output image is minimized by minimizing L2 loss function. For HFFM, we fuse the main processing blocks of 4 heterogeneous deep neural networks in a global network, then connect the output features, and finally input them to the classifier for prediction. SSFE can be trained independently of HFFM with different datasets which make the model have good extensibility. Specifically, this framework naturally support the transfer learning paradism which is widely used in deep learning.

### 2.2. Self-Supervised Patch Encoding Network

SSFE module encodes one patch at a time, and all valid patches of a WSI are encoded and stacked into a feature cube according to their spatial positions. The backbone structure (encoder) of SSFE is similar to that of VGG network. It consists of several connected blocks, each of which consists of a convolution layer, a pooling layer and an activation layer. Supposing that the dimension of the input square patch is *W* × *W* × 3, after passing through the encoder of SSFE, the dimension of the output feature map is *V* × *V* × *K*, where *K* is the channel number of the last convolution layer and *V* < <*W*. A global aggregation pooling is applied to the output feature map, and thus, a 8 × 8 × *K* feature vector is obtained. The reason of applying this pooling operation is twofold. The first is to find the most salient points locally through maximum pooling and introduce an attention mechanism to the model, and the second is to reduce the size of the feature map and improve the processing efficiency of HFFM.

The network structure of SSFE is shown in Figure 2. The red arrow represents the convolution operation with a kernel size of 3 × 3, and the green arrow represents the convolution operation with a kernel size of 1 × 1, which is only used for the output layer of the last decoder. And the yellow arrow represents the maximum pooling or upsampling operation. The yellow block represents the feature map duplication, which is widely used in UNet architecture to image reconstruction and expression of key features. The number above each block (green or yellow) indicates the number of channels of the feature map at this stage. As can be seen from the figure, the feature map size decreases as it goes down, but the number of channels increases. The nonlinear activation layer is not shown in Figure 2. We use the ReLU function [33] here as its effectiveness has been widely verified.

The article "High-Resolution Histopathological Image Classification Model Based on Fused Heterogeneous Networks with Self-Supervised Feature Representation" was published in 2022. Journal: Biomed Res Int.

The decoder performs upsampling with kernel 2 × 2 and convolution with kernel 3 × 3 to recover the input image. SSFE is trained with L2 loss function evaluating the pixel-wise loss between the input patch and recovered one. The connection between encoder and decoder part of SSFE is established through a feature vector, as shown in the central bottom part of Figure 2. As can be seen visually from Figure 2, the image generated by SSFE can well preserve the structure, color, and texture of the original image. The hidden layers of SSFE generate compact feature representations of an input image patch. The reason of choosing the bottom hidden layer for feature representation is that it is the last layer of downsampling, and the length of the feature expression is minimal, while the information of the input patch is retained as much as possible. Thus, the parameter scale of the following classification module can be maintained at a low level.

One of the key problems is that WSIs in a dataset often have different sizes. For example, in TCGALGG dataset, the width of WSI varies between 7949 and 169786 pixels and the height varies between 7152 and 84976 pixels. It results in different number of patches of each WSI after segmentation. The size of feature map in feature cube after SSFE is also different. In order to provide a uniform size feature cube for the later heterogeneous network, an independent layer with fixed parameters is added to reform it.  Figure 3 shows the whole process of generating the feature cube.

Formally, suppose a WSI is divided into *r* rows and *c* columns of nonoverlapping patches in a grid. The feature map of the patch in row *i* and column *j* is *M*^(*ij*)^. In the global average pooling layer, sliding windows are performed on each feature map, the maximum values of sliding windows are obtained, and then, these maximum values are averaged to obtain a feature value representing the feature map. The maximum operation eliminates the influence of local minima on feature value, as shown in

(2) $$\begin{array}{c} v_{ij}=\frac{1}{p\times q}\underset{pq}{\sum }\max\left(sw\left(M_{pq}^{\left(ij\right)}\right)\right), \end{array}$$

where *sw*(*M*_*pq*_^(*ij*)^) returns all values containing in a sliding window centered on point *M*_*pq*_^(*ij*)^.

### 2.3. Fused Heterogeneous Networks

The WSI embedding matrix obtained in the previous section are sent to 4 subnetworks composed of main blocks of heterogeneous networks for training.

#### 2.3.1. Inception Module in GoogleNet

The core idea of GoogleNet [25] is inception module. A number of convolution or pooling operations are put together to assemble an inception module, and the network structure is assembled with the inception module as the unit.  Figure 4 shows the basic structure of an inception module.

The article "High-Resolution Histopathological Image Classification Model Based on Fused Heterogeneous Networks with Self-Supervised Feature Representation" was published in 2022. Journal: Biomed Res Int.

The structure of inception can make full use of computing resources and obtain more effective deep features in the same amount of computation. Therefore, it may improve the classification performance of the entire network. Inspired by network in network [31], 1 × 1 convolutional layer is used in the inception module. There are two main advantages of 1 × 1 convolution operation [31], i.e., cross-channel feature integration and reducing the number of convolution kernel parameters in the model.

#### 2.3.2. VGGNet

The architecture of VGGNet [28] is firstly proposed by Oxford's Visual Geometry Group. The idea of VGGNet is that increasing the depth of the model can affect the final performance to a certain extent. The experimental results on the ImageNet show the effectiveness of VGGNet. Several successive 3 × 3 convolution kernels are used to replace the larger convolution kernel (e.g., 5 × 5, 7 × 7, and 11 × 11) in traditional network (e.g., AlexNet [34]). For convenience of expression, we define VGG block as several stacked 3 × 3 convolution kernels with max pooling and nonlinear activation layers.  Figure 5 shows the architecture of VGGNet.

In VGG, three 3 × 3 convolution kernels are used instead of 7 × 7 convolution kernels, and two 3 × 3 convolution kernels are used instead of 5 × 5 convolution kernels. The main purpose of this design is to improve the depth of the network and the model performance to a certain extent while keeping the same receptive field. The structure of VGGNet is simple, and the convolution kernel (3 × 3) and the maximum pool (2 × 2) are used in the whole network.

#### 2.3.3. Residual Block in ResNet

The core idea of ResNet [29] is to introduce a constant shortcut connection to skip one or more layers directly. It effectively solves the problem of gradient disappearance and explosion of extremely deep network. Specifically, the residual block adopts a structure similar to VGG, but the residual connection is added between two convolution layers. According to [29], the structure of residual block used in this paper is shown in Figure 6.

In Figure 6, the block BN stands for batch normalization and the ⊕ stands for matrix addition. The BN and ReLU layers are carried out before the convolution layer. This preactivation strategy can improve the network performance to a certain extent.

#### 2.3.4. Dense Block in DenseNet

DenseNet got rid of the stereotype thinking of deepening the network layer number and widened the network structure to improve the network performance. It greatly reduced the number of network parameters and alleviated the problem of gradient vanishing through feature reuse and the bypass setting. The input of each layer comes from the output of all previous layers.  Figure 7 shows the architecture of a DenseNet with 3 dense blocks.

The article "High-Resolution Histopathological Image Classification Model Based on Fused Heterogeneous Networks with Self-Supervised Feature Representation" was published in 2022. Journal: Biomed Res Int.

In a dense block, each circle represents a group of operations, including BatchNormalization, ReLU, and convolution. The input of each group is composed of the outputs of all previous layers in the block. The transition layers include a convolution layer and an average pooling layer. The size of the feature map in each block needs to be consistent for connection, and transition layers are inserted between blocks for downsampling operation. DenseNet can accept a small number of feature maps as outputs of the network layer.

#### 2.3.5. Feature Fusion

The feature maps from the four subnetwork are processed by global average pooling and then concatenate to form a feature vector. The feature vectors are input into a dropout layer and a full connection layer, and finally, the predicted category information is output by softmax. Cross entropy loss function and Adam optimizer are used in training.

### 2.4. Model Complexity

Although the WSI processed by this model has ultrahigh resolution, due to the patch-based feature extraction method, there is a linear relationship between the time complexity of SSFE and the number of patches. For a single patch, the training time complexity is comparable to a UNet with an input of 1024 × 1024 × 3. For HFFM, its four subnetworks are stacked by four different types of blocks (see 2.3). The parameter size of each subnetwork is about 1/2 of its reference network, and its training and prediction cost can be evaluated accordingly.

## 3. Evaluations and Results

### 3.1. Dataset and Environment

We evaluated the performance of the proposed model on two public pathological image datasets of TCGA: low grade glioma (LGG) and glioblastoma multiforme (GBM). There are 921 WSI images in the two datasets, which are divided into IDH wild type and mutant. The total size of WSI data used for evaluation exceeds 230 G. We crop the blank part of the image by selecting the smallest circumscribed rectangle containing all tissue areas in the image as effective training area. A set of default filters [35] are applied to each WSI to remove marking pen tracking and small objects. It is worth noting that there are some WSIs containing multiple targets (see Figure 8 for an example). We wrote a script to put each individual target in WSI into a single image. Each WSI is segmented and patches containing effective tissue pixels (no less than 90%) are generated. The patch size is 1024 × 1024 × 3.

The article "High-Resolution Histopathological Image Classification Model Based on Fused Heterogeneous Networks with Self-Supervised Feature Representation" was published in 2022. Journal: Biomed Res Int.

All training and evaluation of the models are carried out on a server with Intel (R) Xeon (R) W2245 CPU @ 3.90 GHz, 64 GB memory, and NVIDIA RTX4000 8 G graphics card. The code for experiment is implemented in Python, and Keras is used for the construction and training of deep neural networks.

### 3.2. Model Setting and Training

SSFE and HFFM are trained separately. For SSFE, the training set is constructed by randomly selecting 600 patches from each dataset. After training, we use the output of the 5th downsampling layer in SSFE as the feature representation for each patch in a WSI. For the sake of improving the model generalization ability, the training dataset is augmented by horizontal and vertical flip. The dimension of extracted feature for each patch is 56 × 56 × 256. And then, a 7 × 7 max pooling is applied to obtain a 8 × 8 × 256 final feature representation. The features extracted through SSFE are placed according to their spatial information to form a WSI embedding matrix as indicated by Figure 3. In order to eliminate the influence of the background on the main part of the image, we perform a threshold operation on the embedding matrix by setting the feature of the patch containing less than 30% of the tissue area with zero. Since the sizes of WSI are not completely consistent, we reform the WSI feature map to make them the same size (56 × 56 × 256) on the premise of keeping the number of channels unchanged.  Figure 9 shows the original and SSFE regenerated patches. It can be seen that the image generated by SSFE can well preserve the structure, color, and texture of the original image.

The whole dataset is divided into training set and test set at the ratio of 9: 1. In the training set, 25% data are randomly selected as the verification set, and the rest 75% are used for model training. The loss function for training SSFE is L2 loss and the optimizer is Adam.

We separately train 4 deep neural networks (VGG, GoogleNet, ResNet, and DenseNet) to classify WSIs represented by features extracted through SSFE. We use these 4 networks as baseline models for comparison with HFFM. They use the same training settings as follows. The batch size is 32 and epoch is 80.

### 3.3. Results

Accuracy (Acc), precision, recall, and F1 score are used for evaluating the performance of all models. These metrics are widely used in measuring the performance of classification models. The definitions are as follows:

(3) $$\begin{array}{c} \text{Acc}=\frac{\text{TP}+\text{TN}}{\text{TP}+\text{TN}+\text{FP}+\text{FN}}, \end{array}$$

(4) $$\begin{array}{c} \text{Precision}=\frac{\text{TP}}{\text{TP}+\text{FP}}, \end{array}$$

(5) $$\begin{array}{c} \text{Recall}=\frac{\text{TP}}{\text{TP}+\text{FP}}, \end{array}$$

(6) $$\begin{array}{c} \text{F}1\text{ score}=\frac{2\times \text{precision}\times \text{recall}}{\text{precision}+\text{recall}}, \end{array}$$

where TP, TN, FP, and FN stand for true positive, true negative, false positive, and false negative, respectively.

The article "High-Resolution Histopathological Image Classification Model Based on Fused Heterogeneous Networks with Self-Supervised Feature Representation" was published in 2022. Journal: Biomed Res Int.

Model 1∼Model 5 represent the use of different subnetwork fusion strategies in HFFM, as shown in Table 1. The classification performance comparison of different models on each metric is shown in Table 2. The last column in Table 2 is the accuracy improvement ratio which represents the improvement of the classification accuracy of the fusion models (*J*) compared to the basic models (*H*), as shown in

(7) $$\begin{array}{c} \text{AccIm}{\text{p}}_{i}=\frac{\left(\text{Ac}{\text{c}}_{i}-\text{Ac}{\text{c}}_{\max H}\right)}{\text{Ac}{\text{c}}_{\max H}}, \end{array}$$

where *Acc*_*i*_ is the classification accuracy of model *i* and Acc_max*H*_ is the maximal classification accuracy of basic models.

It can be seen that the classification performance of the fused networks are greatly improved than those of the basic models. And the model that is fused of all subnetworks achieves the best accuracy among all models. We can see that ResNet and DenseNet have relatively similar classification performance, which is partly caused by similar structures of these two networks.  Figure 10 shows the ROC (receiver operating characteristic) curve of each model and the corresponding AUC (area under ROC) values. It can be seen that Model 5 achieves the highest AUC (0.97) which indicates its best classification performance.

In order to better compare the classification performance between different algorithms, we use Friedman test which was proposed by Milton Friedman in 1937 to evaluate and compare the classification performance of multiple algorithms [36]. The motivation of using Friedman test is twofold. On one hand, it compares the classification performance of different algorithms by calculating the average rank *R* of different datasets in the same algorithm. The smaller value of *R*, the better classification performance of the corresponding algorithm.  Table 3 shows the model ranks. On the other hand, Friedman test can show whether there is significant difference of the models.

From Table 3, it can be seen that Model 5 achieves the lowest rank value 1.0, which is much lower than the rank value of other classification algorithms, indicating the best classification performance of the model. In addition, it can be seen that the rank of VGG and GoogleNet classification networks are 8.0 and 9.0, which are highest among all models. And it can be said that their classification performance is of no significant difference. Model 1, Model 2, and Model 3 have rank values 3.0, 4.0, and 5.0, meaning their almost equal performance on TCGA dataset. Finally, on the whole, the rank of Model 5 is generally 2-8 times smaller than the basic models, which further illustrates the effectiveness of the proposed model.

The article "High-Resolution Histopathological Image Classification Model Based on Fused Heterogeneous Networks with Self-Supervised Feature Representation" was published in 2022. Journal: Biomed Res Int.

## 4. Conclusions

In this paper, we have proposed a novel framework for WSI classification. The framework is composed of a self-supervised feature extraction network and a classification network fused by 4 basic convolutional blocks from heterogeneous network. The self-supervised feature extraction network adopts a UNet-like architecture to extract the deep feature of each patch in a WSI while keeping their spatial information. The extracted features are ensembled in a WSI embedding matrix for classification. Our method achieved an accuracy of 89% on TCGA dataset which outperforms single model, i.e., VGG, GoogleNet, ResNet, and DenseNet, by considerable margins. In addition, compared with the fusion model, our heterogeneous network can also obtain the best classification outcome. Moreover, Friedman test is used to further verify the effectiveness of our model. The rank of the proposed model is 1.0 which is smallest than those of all other models, which proved that our method has significant difference with other models. Future work includes the design of a united network model to process WSIs with different resolutions and magnification, as well as the fusion or ensemble strategy for network blocks with different intuition, e.g., convolution or vision transformer.

## Figures and Tables

**Figure 1:** The main framework of the proposed model.

**Figure 2:** SSFE architecture.

**Figure 3:** Patch encoding

**Figure 4:** Inception module in GoogleNet.

**Figure 5:** The architecture of VGGNet.

**Figure 6:** The architecture of residual block.

**Figure 7:** The architecture of a DenseNet with 3 dense blocks.

**Figure 8:** A WSI containing multiple targets.

**Figure 9:** The original and SSFE generated patches. The first row is original images, and the second row is images generated by SSFE.

**Figure 10:** ROC curves of all models.

**Table 1:** Different subnetwork fusion strategies.

Name	Strategy
Model 1	VGG, ResNet, and DenseNet
Model 2	VGG, GoogleNet, and ResNet
Model 3	VGG, GoogleNet, and DenseNet
Model 4	GoogleNet, ResNet, and DenseNet
Model 5	VGG, GoogleNet, ResNet, and DenseNet

**Table 2:** Classification performance comparison of different models on TCGA dataset.

	Model	Acc	Precision	Recall	F1 score	AccImp
H	VGG	0.790	0.791	0.795	0.789	−
	GoogleNet	0.780	0.812	0.799	0.779	−
	ResNet	0.820	0.827	0.830	0.820	−
	DenseNet	0.820	0.830	0.830	0.820	−

J	Model 1	0.860	0.858	0.863	0.859	4.9%
	Model 2	0.840	0.840	0.845	0.839	2.4%
	Model 3	0.850	0.848	0.847	0.847	3.7%
	Model 4	0.880	0.883	0.873	0.877	7.3%
	Model 5	0.890	0.889	0.887	0.888	8.5%

The article "High-Resolution Histopathological Image Classification Model Based on Fused Heterogeneous Networks with Self-Supervised Feature Representation" was published in 2022. Journal: Biomed Res Int.

**Table 3:** Model ranks.

Model	Rank	Model	Rank
Model 1	3.0	VGG	8.0
Model 2	5.0	GoogleNet	9.0
Model 3	4.0	ResNet	6.5
Model 4	2.0	DenseNet	6.5
Model 5	1.0		

## Data Availability

The WSI data used to support the findings of this study have been deposited in the TCGA repository (https://www.cancer.gov/about-nci/organization/ccg/research/structural-genomics/tcga).
